# Alterations in mGluR5 Expression and Signaling in Lewy Body Disease and in Transgenic Models of Alpha-Synucleinopathy – Implications for Excitotoxicity

This article has been retracted.

**DOI:** 10.1371/journal.pone.0014020

**Published:** 2010-11-16

**Authors:** Diana L. Price, Edward Rockenstein, Kiren Ubhi, Van Phung, Natalie MacLean-Lewis, David Askay, Anna Cartier, Brian Spencer, Christina Patrick, Paula Desplats, Mark H. Ellisman, Eliezer Masliah

**Affiliations:** 1 Department of Neurosciences, University of California San Diego, La Jolla, California, United States of America; 2 Department of Pathology, University of California San Diego, La Jolla, California, United States of America; 3 National Center for Microscopy and Imaging Research, University of California San Diego, La Jolla, California, United States of America; 4 Center for Research in Biological Systems, University of California San Diego, La Jolla, California, United States of America; Tokyo Medical and Dental University, Japan

## Abstract

Dementia with Lewy bodies (DLB) and Parkinson's Disease (PD) are neurodegenerative disorders of the aging population characterized by the abnormal accumulation of alpha-synuclein (alpha-syn). Previous studies have suggested that excitotoxicity may contribute to neurodegeneration in these disorders, however the underlying mechanisms and their relationship to alpha-syn remain unclear. For this study we proposed that accumulation of alpha-syn might result in alterations in metabotropic glutamate receptors (mGluR), particularly mGluR5 which has been linked to deficits in murine models of PD. In this context, levels of mGluR5 were analyzed in the brains of PD and DLB human cases and alpha-syn transgenic (tg) mice and compared to age-matched, unimpaired controls, we report a 40% increase in the levels of mGluR5 and beta-arrestin immunoreactivity in the frontal cortex, hippocampus and putamen in DLB cases and in the putamen in PD cases. In the hippocampus, mGluR5 was more abundant in the CA3 region and co-localized with alpha-syn aggregates. Similarly, in the hippocampus and basal ganglia of alpha-syn tg mice, levels of mGluR5 were increased and mGluR5 and alpha-syn were co-localized and co-immunoprecipated, suggesting that alpha-syn interferes with mGluR5 trafficking. The increased levels of mGluR5 were accompanied by a concomitant increase in the activation of downstream signaling components including ERK, Elk-1 and CREB. Consistent with the increased accumulation of alpha-syn and alterations in mGluR5 in cognitive- and motor-associated brain regions, these mice displayed impaired performance in the water maze and pole test, these behavioral alterations were reversed with the mGluR5 antagonist, MPEP. Taken together the results from study suggest that mGluR5 may directly interact with alpha-syn resulting in its over activation and that this over activation may contribute to excitotoxic cell death in select neuronal regions. These results highlight the therapeutic importance of mGluR5 antagonists in alpha-synucleinopathies.

## Introduction

Movement disorders with parkinsonism and cognitive impairment continue to be a significant neurological problem in the aging population. While patients with classical Parkinson's Disease (PD) present with tremor, motor deficits and autonomic dysfunction(s), others patients develop cognitive alterations including dementia. Patients that present first with cognitive impairments followed by development of parkinsonism are denominated dementia with Lewy bodies (DLB) to distinguish them from patients with PD dementia (PDD). Jointly this heterogeneous group of disorders is referred to as Lewy body disease (LBD) [1]. These conditions are associated with progressive and selective loss of dopaminergic and non-dopaminergic cells [2] and the formation of Lewy bodies (LBs) and Lewy neurites containing fibrillar alpha-synuclein (alpha-syn) [3], [4], [5], [6], [7], [8] in cortical and subcortical regions [9], [10], [11]. Previous studies have suggested that excitotoxicity may contribute to neurodegeneration in these disorders however the underlying mechanisms and their relationship to alpha-syn remain unclear.

Synucleins are a family of related proteins including alpha-, beta-, and gamma-synuclein. Alpha-syn is a 14 kDa 'naturally unfolded protein' [12], [13] abundant at the presynaptic terminal [14] and likely plays a role in modulating vesicular synaptic release [15]. Abnormal accumulation of alpha-syn is thought to be centrally involved in the pathogenesis of both sporadic and inherited forms of parkinsonism as mutations and multiplications in the alpha-syn gene have been associated with rare familial forms of PD [4], [8], [16]. In addition, over expression of alpha-syn in transgenic (tg) mice [17], [18], [19] and *Drosophila* [20] recreates several pathological and dysfunctional motor performance features of PD. Recent studies have shown that accumulation of oligomeric, rather than polymeric (fibrilar) forms of alpha-syn in the synapses and axons may be responsible for neuronal dysfunction and degeneration [21], [22], [23].

In addition to the modulation of vesicular synaptic release, alpha-syn has been shown to regulate dopaminergic neurotransmission (reviewed by [24]) and to be involved in dopamine release [25], [26] whilst dopamine in turn, has been reported to promote alpha-syn oligomerization [27], [28]. These interactions between dopamine and alpha-syn may help explain the selective vulnerability of the dopaminergic system in PD. Recent studies have demonstrated that, in addition to well-documented dopaminergic alterations, other neurotransmitter systems are also dysregulated in PD and DLB. For example, altered glutamatergic neurotransmission within basal ganglia circuitry is thought to contribute to the clinical presentation of parkinsonian-related motor symptoms, though the mechanisms underlying this are not yet fully understood. Abnormal activation of group I metabotropic receptors (mGluR1 and mGluR5) within the basal ganglia circuitry has been proposed to account for cognitive and motor alterations in patients with DLB [29], [30], [31]. mGluR5 in particular has attracted considerable interest because of its potential involvement in Alzheimer's Disease (AD) [32] and PD [33], [34], its role in learning and memory [35], [36], and its abundant expression in the frontal cortex, limbic system, and caudoputamen [37]—brain regions selectively affected in AD and PD.

Further support for a role of group I mGluR receptors in the pathogenesis of PD and DLB steams from studies showing that mGluR5 antagonists ameliorate the behavioral alterations in animal model of parkinsonism [38], [39], [40], [41] and are neuroprotective against MPTP (1-methyl-4-phenyl-1,2,3,6-tetrahydropyridine) neurotoxicity in animals [42], [43]. Mice lacking the mGluR5 receptors also display reduced MPTP toxicity [43].

Although extensive behavioral pharmacology studies with mGluR5 antagonists in PD-like animal models have been performed, surprisingly very limited information is available as to the potential role of alterations in mGluR's in the pathogenesis of the excitotoxicity in PD or DLB patients, or alpha-syn tg animal models. Here we describe studies of mGluR5 expression the brains of patients with DLB or PD and in alpha-syn over-expressing tg mice, and discuss a role for altered mGluR5 expression in excitotoxicity. Furthermore, we present evidence that mGluR5 receptor antagonism is capable of ameliorating the behavioral deficits observed in alpha-syn tg mice. Taken together these results support the notion that mGluRs play an important role in the pathogenesis of disorders with alpha-syn accumulation and that mGluR5 receptors may be an important target for therapeutic intervention.

## Materials and Methods

### Human specimens, Neuropathological Evaluation and Criteria for diagnosis

A total of 24 cases (n = 8 non-demented controls; n = 8 DLB and n = 8 PD cases) were included for the present study. Autopsy material was obtained from patients (Table 1) studied neurologically and psychometrically at the Alzheimer Disease Research Center/University of California, San Diego (ADRC/UCSD). The last neurobehavioral evaluation was performed within 12 months before death and included Blessed score, Mini Mental State Examination (MMSE) and dementia-rating scale (DRS) [44], [45]. Brains were processed and evaluated according to standard methods [46]. At autopsy, brains were divided sagitally, the left hemibrain was fixed in formalin of 4% paraformaldehyde (PFA) for neuropathological analysis and the right frozen at −70°C for subsequent neurochemical analysis. Paraffin sections from 10% buffered formalin-fixed neocortical, limbic system and subcortical material stained with hematoxylin and eosin (H&E), thioflavine-S, ubiquitin (Dako, Carpinteria, CA) and α-syn (Millipore, Temecula, CA) were used for routine neuropathological analysis that included assessment of plaques, tangles, Lewy bodies and Braak stage [46]. The diagnosis of DLB was based in the initial clinical presentation with dementia followed by parkinsonism and the presence of alpha-syn and ubiquitin-positive LBs in cortical and subcortical regions [47], [48]. The diagnosis of PD was based on the initial presentation with parkinsonism and presence of alpha-syn and ubiquitin positive LBs in subcortical regions.

**Table 1:** Summary of clinical neurobehavioral and post-mortem features for human samples.

Group	N	Age(years, mean ± SEM)	GenderM/F	PMT(hours, mean ± SEM)	Braak stage	Blessed score(mean ± SEM)	Brain weight (grams, mean ± SEM)	LBs neocortex(score)	LBs midbrain(score)
Control	8	76 (±10)	2/3	8 (±3)	0	0	1200 (±97)	0	0
Dementia with Lewy bodies	8	83 (±5)	4/1	9 (±2)	III-IV	28 (±3)	1216 (±85)	3+	2+
Parkinson's Disease	8	77 (±8)	3/2	6 (±2)	0	5 (±2)	1276 (±128)	0	3+

LBs =  Lewy bodies; PMT =  postmortem time, SEM  =  standard error of the mean.

### Transgenic mouse lines

Transgenic mice over expressing wildtype human (h) alpha-syn under the control of the platelet-derived growth factor (PDGF) (D-line; [19]) and the mThy1 (line 61; [49]) promoters were used. The PDGF-alpha-syn tg mice were selected because they display accumulation of α-syn in the frontal cortex and limbic system similar to DLB accompanied by behavioral deficits, early motor alterations, loss of dopaminergic terminals and formation of inclusion bodies [19]. The mThy1-alpha-syn tg mice were selected because they display more extensive α-syn accumulation in the frontal cortex, limbic system and subcortical regions including the basal ganglia and the substantia nigra. For the immunoblot and immunochemical studies a total of 24 mice were used (n = 8 non-tg; n = 8 PDGF-alpha-syn and n = 8 mThy1-alpha-syn tg) age 6 months old. For the behavioral and therapeutic studies a total of 36 animals were utilized (n = 12 non-tg; n = 12 PDGF-alpha-syn and n = 12 mThy1-alpha-syn tg) at 9 months of age. From each of the groups half of the mice (n = 6) were treated with vehicle only and the other half (n = 6) were treated with MPEP (2-Methyl-6-(phenylethynyl)-pyridine).

### Treatment with mGluR5 antagonist and Behavioral testing

For these experiments MPEP, a selective and systemically active mGluR5 receptor antagonist, was used to test the effects of mGluR5 receptor antagonism on behavioral performance [50]. MPEP HCl was obtained from Tocris Biosciences (Ellisville, MO; Catalog #1212), and dissolved in 0.9% saline solution at a dose of 20 mg/ml. This dose was chosen based on reports in the literature demonstrating effective dose ranges for behavioral studies in mice without adverse effects [51], [52]. The MPEP solution was sonicated to ensure complete dilution and the solution was used the same day. MPEP was administered by intraperitoneal (IP) injection, the animals were weighed on the day of testing and the appropriate volume was determined and recorded for each animal (approximately 0.2 ml/animal). A 30-minute pre-injection time was used, and administration times were staggered to account for this time prior to testing. The behavioral effects of MPEP in the α-syn over-expressing tg mice were tested in the vertical pole test (motor test) and the Morris water maze (learning and memory test).

The pole test was divided into 3 phases, including a pretest (with saline injection), a challenge with MPEP administration, and a reassessment (no injections) to determine performance one week after MPEP administration. The percentage change in performance from Test 1 to Test 2 was determined by calculating the difference between success ratios on these two separate test days. Animals underwent testing on a vertical pole apparatus to evaluate their ability to negotiate and descend the apparatus. The testing procedures were derived from previous reports [53], [54]. The apparatus consists of a rough-surfaced pole (diameter 1 cm; height 50 cm) inserted perpendicular to a circular platform. The pole was lightly roughened with medium grade sandpaper in between animals to ensure that all animals were presented with a comparable pole surface. The circular platform was covered with multilayered padding to avoid injury to the animals in the event of a fall from the apparatus. The top padded surface was disposable and frequently changed to avoid a soiled surface. Non-tg mice easily complete this task, and to date, our group has noted performance deficits in the alpha-syn tg mice as early as 4 months of age. The pole testing session consisted of 2 training trials followed by 5 test trials (7 trials total). The first 2 untimed trials served to acquaint the animal with the apparatus. The 5 test trials were timed to a maximum of 120 sec. Two timed measures were recorded including: (1) the time until the animal completely turned around and re-oriented towards platform base (T-Turn), and (2) the total time spent on apparatus (T-Total). This procedure was repeated a total of 5 times. The ratio of success for each subject based on the number of times (out of 5 total trials) the apparatus was successfully negotiated was noted.

To evaluate the effects of MPEP on learning and memory in the alpha-syn over-expressing tg mice they were tested in the Morris water maze as previously described [55]. Mice were treated for 28 days with saline vehicle solution of MPEP as a daily IP injection (20 mg/ml, 0.2 ml per animal per day). At day 20 of the treatments mice were tested in the water maze for 8 days. For this purpose a pool (diameter 180 cm) was filled with opaque water (24°C) and mice were first trained to locate a visible platform (days 1–3) and then a submerged hidden platform (days 4–7) in three daily trials 2–3 min apart. Mice that failed to find the hidden platform within 90 seconds were placed on it for 30 seconds. The same platform location was used for all sessions and all mice. The starting point at which each mouse was placed into the water was changed randomly between two alternative entry points located at a similar distance from the platform. On day 7, another visible platform trial was performed to exclude differences in motivation and fatigue. On day 8 the platform was removed (probe test) and mice were tested to evaluate the numbers of entrances and time expended in the target quadrant. Time to reach the platform (latency), path length, and swim speed were recorded with a Noldus Instruments EthoVision video tracking system (San Diego Instruments, San Diego, CA) set to analyze two samples per second. UCSD is an Institutional Animal Care and Use Committee accredited institution and the UCSD Animal Subjects Committee approved the experimental protocol followed in all studies according to the Association for Assessment and Accreditation of Laboratory Animal Care International guidelines.

### Immunoblot analysis

The immunoblot procedures for human and transgenic mouse samples were performed as previously described [19]. Briefly, dissected frozen tissues were homogenized, and processed and separated into cytosolic and particulate fractions. The nuclear fraction was obtained by resuspending the pellet (from the 5000 g spin after homogenization) in buffer +1%SDS +1% TritonX. Incubated on ice for 15 minutes, vortexing every 3 minutes, then centrifuged for 10 minutes at 14,000 g at 4°C. The protein concentrations of individual samples were determined using a BCA protein assay kit (Pierce Biotechnology, Rockford, IL). Approximately 20 ug of each fraction were loaded onto either 3–8% Tris-acetate (mGluR5 human) or 4–12% Bis-Tris (all others) SDS polyacrylamide gel electrophoresis (SDS/PAGE) gels (Invitrogen, Carlsbad, CA), transferred into Immobilon membranes (Millipore, Temecula, CA), blocked with either 3% BSA (for animal samples) or 5% Milk/1% BSA (for human samples) in PBS, and incubated overnight at 4°C with antibodies against mGluR5 (rabbit polyclonal, 1∶1000, Millipore, Temecula, CA), beta-arrestin (rabbit polyclonal, 1∶1000, Cell Signaling, Boston, MA), extracellular signal-regulated kinase (ERK, mouse monoclonal, 1∶1000, Cell Signaling, Boston, MA), phospho-ERK (pERK, mouse monoclonal, 1∶1000 Cell Signaling, Boston, MA), Elk-1 member of ETS oncogene family (Elk-1, rabbit polyclonal, 1∶1000, Cell Signaling, Boston, MA, phospho-Elk-1 (pElk-1, rabbit polyclonal, 1∶1000, Cell Signalling, Boston, MA), cAMP response element-binding (CREB, mouse monoclonal, 1∶1000 Cell Signaling, Boston, MA) and phospho-CREB (pCREB, rabbit polyclonal, 1∶1000 Cell Signaling, Boston, MA). The next day, blots were rinsed several times and incubated with the appropriate secondary antibody on a shaker for 1 hour at room temperature. Membranes were processed using a chemiluminescence kit (Western Lightning Chemiluminescence Reagent Plus; Perkin Elmer, Boston, MA) and imaged using a Versadoc system (Biorad, Hercules, CA). Following imaging, the membranes were processed for further immunolabeling using an antibody re-probing kit (Chemicon, Temecula, CA). Actin loads (Beta-actin, mouse monoclonal, Sigma, St. Louis, MO) were then determined for each membrane as a control for protein loading. All mGluR5 protein levels were normalized using the actin immunoreactivity values. The Quality One™ image analysis program (Biorad, Hercules, CA) was used for quantitative assessment of bands. Statistical analyses were performed using one-way ANOVAs and the level for significance set at p<0.05. Resultant data were graphed using SigmaPlot 9.0 (Systat Software Inc., Richmond, CA). Graphed data are presented as the mean optical density (group means mGluR5/actin immunolevels) ± the standard error of the mean (SEM).

### Tissue processing, immunocytochemical analysis and laser scanning confocal microsocopy

Briefly, as previously described [56], free-floating 40 µm thick vibratome sections were washed with Tris buffered saline (TBS, pH 7.4), pre-treated in 3% H2O2, and blocked with 10% serum (Vector Laboratories, Burlingame, CA), 3% bovine serum albumin (Sigma), and 0.2% gelatin in TBS-Tween (TBS-T). For human brains, sections from the frontal cortex, hippocampus and putamen were used; for the mice sagittal sections from the complete brain were studied. Sections were incubated at 4°C overnight with the monoclonal antibodies against mGluR5 (Millipore) and beta-arrestin (Cell Signaling) or the polyclonal antibody against α-syn (Millipore). Sectionswere then incubated in secondary antibody (1∶75, Vector), followed by Avidin D horseradish peroxidase (HRP, ABC Elite, Vector) and reacted with diaminobenzidine (DAB, 0.2 mg/ml) in 50 mM Tris (pH 7.4) with 0.001% H_2_O_2_. Control experiments consisted of incubation with pre-immune rabbit serum. To investigate the effects of postmortem delay and fixation on the levels of mGluR5 immunoreactivity, preliminary studies were performed in a subset of cases (n = 5) with postmortem delay ranging from 4–48 h. Immunostained sections were imaged with a digital Olympus microscope and assessment of levels of mGluR5 and arrestin immunoreactivity was performed utilizing the Image-Pro Plus program (Media Cybernetics, Silver Spring, MD). For each case a total of three sections (10 digital images per section at 400x) were analyzed in order to estimate the average number of immunolabeled cells per unit area (mm^2^) and the average intensity of the immunostaining (corrected optical density).

Double-immunocytochemical analyses was performed utilizing the Tyramide Signal Amplification™-Direct (Red) system (NEN Life Sciences, Boston, MA) to detect alpha-syn. Specificity of this system was tested by deleting each primary antibody. For this purpose, sections were double-labeled with the monoclonal antibodies against alpha-syn (1∶20,000, Millipore) detected with Tyramide Red, and mGluR5 detected with fluorescein isothiocyanate (FITC)-conjugated secondary antibodies (1∶75, Vector). All sections were processed simultaneously under the same conditions and experiments were performed twice for reproducibility. Sections were imaged with laser scanning confocal microscope BioRad Radiance 2000 (Hercules, CA) equipped with a Nikon E600FN Ellipse microscope (Japan) and using a Nikon Plan Apo 60x oil objective (NA 1.4; oil immersion).

### Tissue section acquisition and immunocytochemistry for large scale mosaic

An additional group of non-tg and PDGF- alpha-syn tg mice (n = 6 per group; 6 month old) were deeply anesthetized with Nembutal™ (pentobarbital) and perfused via intracardiac catheterization. Perfusion with oxygenated Ringer's solution containing 250 U/ml heparin, 0.2 mg/ml xylocaine and 1% dextrose was followed 4% paraformadehyde in 0.1 M phosphate buffer solution (PBS) (both at 37 degrees Celsius). The brains were carefully removed from the skull and postfixed for 1 hour in the same fixative used in the perfusion. The brain was blocked and cut into 2 mm thick sections using an acrylic brain matrix (David Kopf; Tujunga, CA) to facilitate reproducibility of sections. These thick sections were then sectioned into 80 micron thick coronal sections using a Vibratome (VT1000E, Leica Microsystems, Wetzlar, Germany).

Tissue sections were incubated with monoclonal anti-α-syn (1∶250; BD Transduction Laboratories, San Diego, CA) and rabbit anti-mGluR5 (1∶250; Millipore, Temecula, CA) followed by incubation with donkey anti-mouse Alexa Red (1∶100, Molecular Probes, Carlsbad, CA) and donkey anti-rabbit FITC (1∶100, Jackson Immunoresearch Laboratories, Inc., West Grove, PA, USA) overnight at 4C. The immunolabeling procedure consisted of the following steps: (1) 6×5 min rinses in 0.1 M PBS; (2) 1 hr blocking step in PBS containing 3% normal donkey (NDS), 0.1% Triton X-100, 1% fish gelatin, and 1% BSA; (3) 48 hr incubation in primary antibodies diluted in working buffer (PBS, 1% NDS) at 20 degrees C; (4) 6×5 minute rinsed in working buffer; (5) 24 hr incubation in working buffer containing donkey anti-mouse Alexa Fluor 488 (Molecular Probes, Carlsbad, CA) and donkey anti-rabbit RRX (Jackson Immunoresearch Laboratories, Inc., West Grove, PA, USA). (6) 6×10 min rinses in working buffer; (7) 3×10 min rinses in PBS; (8) the sections were free floated onto slides and coverslipped using ProLong mounting media (Invitrogen Molecular Probes, Carlsbad, CA) with DAPI nuclear stain. Controls for the mGluR5 antibody experiments included both preabsorption with the control peptide (Chemicon,Temecula, CA), as well as primary omission studies, which both revealed a lack of non-specific staining (data not shown). Controls for other antibodies used were performed via omission of primary antibodies, and revealed no non-specific staining (data not shown). All steps were conducted at 4°C, on wet ice and with ice-cold solutions.

### Acquisition of large-scale mosaic survey images

The wide-field mosaic image data sets were acquired with the multiphoton scanning system described previously [57], [58] and these were used to survey brain regions for further targeted imaging and analyses. For these purpose, sections double labeled with antibodies against mGluR5 and α-syn as described above were used. Representative large scale images were acquired using a customized video-rate multiphoton microscope [59] equipped with a custom automated high precision motorized stage (Applied Precision LLC, Issaquah, WA), which allows for the automatic acquisition of ultra-large field image mosaics in 2 and 3 dimensions [57], [58]. A Nikon Plan Apo TIRF (60×1.45) oil immersion objective was used. These mosaic images are acquired by rastering the specimen along the X, Y, and Z axes, introducing a prescribed amount of overlap between acquired images (in this case 10%) to aid alignment. Unprocessed image data acquired on the high-speed multiphoton microscope is subsequently stored as a single stack of images. The image stack is analyzed using the JAVA-based ImageJ, a freely available software package, using plugins developed at NCMIR for processing, aligning, and assembling these massive datasets. Briefly, each file is separated into three separate.tiff stacks, one for each channel. Each tile of the image mosaic is normalized to eliminate shading gradients, followed by the automatic alignment of individual tiles to form a full size mosaic image of the data for each channel. A “globally optimized,” normalized cross-correlation algorithm is used to achieve sub-pixel alignment accuracy. The assembled mosaics are then combined into one full-scale color image. For 3D imaging, the process is repeated for each wide field image plane in Z. The large-scale images were used to identify regions of interest for confocal imaging studies.

### Statistical analyses

One-way ANOVAs were performed for water maze and pole test data using the Statview statistical package (version 5.0.1, Cary, NC). Behavioral and image data were graphed using SigmaPlot 9.0 (Systat Software Inc., Richmond, CA). All data are presented as the mean group value ± the standard error of the mean. The criterion for significance was set at p<0.05.

## Results

### Regionally selective increases in the levels of mGluR5 in DLB and PD cases

Given the abundant expression of mGluR5 in brain regions involved in AD and PD such as the frontal cortex, limbic system, and caudoputamen [37], it has been proposed that alterations in mGluR5 may be involved in the pathogenesis of AD [32] and PD [33], [34], [35], [36]. Nonetheless the relative levels of mGluR5 expression and alterations in DLB or PD have not been studied. For this purpose, patterns of distribution for mGluR5 and the downstream regulators were evaluated by immunocytochemistry and immunoblot analysis.

mGluR5 immunoreactivity was associated with pyramidal neurons in layers 2–3 of the frontal cortex (Figure 1), in pyramidal neurons in the CA3 region of the hippocampus and in mid-spiny neurons in the caudo-putamen (Figure S1). Compared to control cases, in DLB there was a significant increase in the levels of mGluR5 immunoreactivity in neurons in the frontal cortex (Figure 1A, B, D), hippocampus (Figure S1, A, B, D) and caudo-putamen region (Figure S1E, F, analyzed in H) Compared to controls, in the PD cases, levels of mGluR5 were increased in the caudo-putamen (Figure S1E, G, H). However levels in the frontal cortex and hippocampus were comparable to controls (frontal cortex, Figure 1A, C, D; hippocampus, Figure S1A, C, D). Beta-arrestin is a downstream regulator of mGluR5 recycling. Group I mGluRs undergo rapid internalization after agonist exposure, this internalization is strongly inhibited by the expression of both beta-arrestin and dynamin dominant-negative mutants [60], [61], [62]. Similar to mGluR5, beta-arrestin was associated with pyramidal neurons in layers 2–3 of the frontal cortex (Figure 1). Compared to controls, beta-arrestin immunoreactivity was increased in the DLB cases in the frontal cortex (Figure 1E, F, H). Compared to controls, PD cases displayed no differences in beta-arrestin immunoreactivity in the frontal cortex (Figure 1E, G, H). As expected, compared to control cases, neocortical alpha-syn levels were much higher in DLB and were associated with LBs in these cases as opposed to the neuritic, punctate staining observed in the controls (Figure 1I, J, L). There was no significant difference in neocortical alpha-syn immunoreactivity in the PD cases compared to controls (Figure 1I, K, L).

**Figure 1:** Immunohistochemical analysis of mGluR5, beta-arrestin and alpha-syn in the frontal cortex of Control, DLB and PD cases. (A, B, C) Representative bright field microscopy images of mGluR5 immunoreactivity in the frontal cortex of control, DLB and PD cases respectively. (D) Analysis of mGluR5 immunoreactivity in the frontal cortex of control, DLB and PD cases. (E, F, G) Representative bright field microscopy images of beta-arrestin immunoreactivity in the frontal cortex of control, DLB and PD cases respectively. (H) Analysis of beta-arrestin immunoreactivity in the frontal cortex of control, DLB and PD cases. (I, J, K) Representative bright field microscopy images of alpha-syn immunoreactivity in the frontal cortex of control, DLB and PD cases respectively. (L) Analysis of alpha-syn immunoreactivity in the frontal cortex control, DLB and PD cases. Scale bar  = 30 µM. * Indicates a significant difference between DLB or PD cases compared to control cases (p<0.05, one-way ANOVA and post hoc Fisher). # Indicates a significant difference between DLB and PD cases (p<0.05, one-way ANOVA and post hoc Fisher) (n = 8 cases per group).

By immunoblot analysis, mGluR5 was identified in the membrane fractions from athe frontal cortex, hippocampus and caudate of controls, DLB and PD cases as a double band with an approximate MW of 132 kDa (Figure 2A, C and E). Compared to controls, in the DLB cases, there was a significant increase in mGluR5 levels in the membrane fractions from the frontal cortex (Figure 2A, B), hippocampus (Figure 2C, D) and caudo-putamen (Figure 2E, F). In PD cases, there was an increase in the levels of mGluR5 in the membrane fraction of the caudo-putamen (Figure 2E, F), but levels in the frontal cortex and hippocampus were comparable to controls (Figure 2A–D). No mGluR5 was detected in the cytosolic fractions. In a subset of the PD cases there appeared to be an inverse relationship between monomeric alpha-syn and mGluR5 levels in the membrane fraction from the frontal cortex. This might be driven by the increased oligomerization of alpha-syn in these cases, which might correlate with the increase of mGluR5. Beta-arrestin was identified as a double band both in the membrane (Figure 2A, C and E) and cytosolic (Figure 2G, I, K) fractions with an approximate MW of 50 kDa. Compared to controls, in the DLB cases, there was a significant increase in beta-arrestin levels in the membrane fractions from frontal cortex (Figure 2A, B), hippocampus (Figure 2C, D) and caudo-putamen (Figure 2E, F). In PD cases, compared to controls, there was an increase in the levels of beta-arrestin in the membrane fractions from the hippocampus (Figure 2C, D) and caudo-putamen (Figure 2E, F), but levels in the frontal cortex were comparable to controls (Figure 2A, B). In the cytoplasmic fractions from the frontal cortex beta-arrestin levels were reduced in both DLB and PD cases compared to controls (Figure 2G, H). In cytoplasmic fractions from the hippocampus, beta-arrestin levels were increased in both DLB and PD cases compared to controls (Figure 2I, J). In cytoplasmic fractions from the caudo-putamen region beta-arrestin levels, in comparison to controls, were unchanged in DLB, but higher in the PD cases (Figure 2K, L).

**Figure 2:** mGluR5, beta-arrestin and alpha-syn expression in frontal cortex, hippocampus and caudate of Control, DLB and PD cases. (A) Representative immunoblot of mGluR5, beta-arrestin and alpha-syn expression levels in the membrane fraction of the frontal cortex from control, DLB and PD cases. (B) Analysis of mGluR5 and beta-arrestin levels in the membrane fraction of the frontal cortex. (C) Representative immunoblot of mGluR5, beta-arrestin and alpha-syn expression levels in the membrane fraction of the hippocampus from control, DLB and PD cases. (D) Analysis of mGluR5 and beta-arrestin levels in the membrane fraction of the hippocampus. (E) Representative immunoblot of mGluR5, beta-arrestin and alpha-syn expression levels in the membrane fraction of the caudate from control, DLB and PD cases. (F) Analysis of mGluR5 and beta-arrestin levels in the membrane fraction of the caudate. (G) Representative immunoblot of mGluR5, beta-arrestin and alpha-syn expression levels in the cytosolic fraction of the frontal cortex from control, DLB and PD cases. (H) Analysis of mGluR5 and beta-arrestin levels in the cytosolic fraction of the frontal cortex. (I) Representative immunoblot of mGluR5, beta-arrestin and alpha-syn expression levels in the cytosolic fraction of the hippocampus from control, DLB and PD cases. (J) Analysis of mGluR5 and beta-arrestin levels in the cytosolic fraction of the hippocampus. (K) Representative immunoblot of mGluR5, beta-arrestin and alpha-syn expression levels in the cytosolic fraction of the caudate from control, DLB and PD cases. (L) Analysis of mGluR5 and beta-arrestin levels in the cytosolic fraction of the caudate. * Indicates a significant difference between DLB or PD cases compared to control cases (p<0.05, one-way ANOVA and post hoc Fisher). # Indicates a significant difference between DLB and PD cases (p<0.05, one-way ANOVA and post hoc Fisher).

### Levels of mGluR5 immunolabeling are elevated in the brains of α-syn transgenic mice

Two different lines of tg mice were used, the first express alpha-syn under the PDGF promoter which favors alpha-syn accumulation in the frontal cortex and limbic system with a distributions similar to DLB. The second express alpha-syn under the mThy-1 promoter, which results in greater accumulation of alpha-syn in subcortical nuclei including the basal ganglia and midbrain, analogous to PD. In both non-tg and tg mice lines, mGluR5 immunoreactivity was associated with pyramidal neurons in layers 2–3 of the frontal cortex (Figure 3A–C), in pyramidal neurons in the CA3 region of the hippocampus (Figure S2A–C) and mid-spiny neurons in the caudo-putamen (Figure S2E–G). Compared to non-tg mice, in PDGF-alpha-syn tg mice there was a significant increase in the levels of mGluR5 immunoreactivity in neurons in the frontal cortex (Figure 3A, B, D), hippocampus (Figure S2A, B, D) and caudo-putamen (Figure S2E, F, H). In the mThy1-alpha-syn tg mice levels of mGluR5 immunoreactivity were similarly increased in the frontal cortex (Figure 3A, C, D), hippocampus (Figure S2A, C, D) and caudo-putamen (Figure S2E, G, H). In the control non-tg mice mild levels of beta-arrestin immunoreactivity were detected in pyramidal neurons in layers 2–3 and 5 of the frontal cortex (Figure 3E). Levels of beta-arrestin immunoreactivity were increased in the frontal cortex of PDGF- and mThy1-alpha-syn tg mice, compared to non-tg mice (Figure 3E–H).

**Figure 3:** Immunohistochemical Analysis of mGluR5, beta-arrestin and alpha-syn in the frontal cortex of alpha-syn transgenic mice. (A, B, C) Representative bright field microscopy images of mGluR5 immunoreactivity in the frontal cortex of non-tg, PDGF-alpha-syn and mThy1-alpha-syn tg mice, respectively. (D) Analysis of mGluR5 immunoreactivity in the frontal cortex of non-tg, PDGF-alpha-syn and mThy1-alpha-syn tg mice. (E, F, G) Representative bright field microscopy images of beta-arrestin immunoreactivity in the frontal cortex of non-tg, PDGF-alpha-syn and mThy1-alpha-syn tg mice, respectively. (H) Analysis of beta-arrestin immunoreactivity in the frontal cortex of non-tg, PDGF-alpha-syn and mThy1-alpha-syn tg mice. (I, J, K) Representative bright field microscopy images of alpha-syn immunoreactivity in the frontal cortex of non-tg, PDGF-alpha-syn and mThy1-alpha-syn tg mice, respectively. (L) Analysis of alpha-syn immunoreactivity in the frontal cortex of non-tg, PDGF-alpha-syn and mThy1-alpha-syn tg mice. Scale bar  = 30 µM. * Indicates a significant difference between alpha-syn tg mice compared to non-tg controls (p<0.05, one-way ANOVA and post hoc Fisher) (n = 8 cases per group).

By immunoblot analysis, mGluR5 was detected in the membrane (Figure 4A) and cytosolic (Figure 4B) fractions as a doublet with an estimated MW of 132 kDa. Consistent with the immunocytochemical studies, levels of mGluR5 in the frontal cortex were elevated in the membrane fractions of the alpha-syn tg mice compared to non-tg controls (Figure 4A, C). Beta-arrestin was detected as a single band at 50 kDa in both the cytosolic and membrane fractions. Compared to non-tg controls, in the PDGF- and mThy1-alpha-syn tg mice the levels of beta-arrestin immunoreactivity were increased the neocotex in both the membrane (Figure 4A, C) and cytoplasmic (Figure 4B, D) fractions.

**Figure 4:** mGluR5, beta-arrestin and alpha-syn expression in frontal cortex of alpha-syn transgenic mice. (A) Representative immunoblot of mGluR5, beta-arrestin and alpha-syn expression levels in the membrane fraction of the frontal cortex from non-tg, PDGF-alpha-syn and mThy1-alpha-syn tg mice. (B) Representative immunoblot of mGluR5, beta-arrestin and alpha-syn expression levels in the cytoplasmic fraction of the frontal cortex from non-tg, PDGF-alpha-syn and mThy1-alpha-syn tg mice. (C) Analysis of mGluR5 and beta-arrestin levels in the membrane fraction of the frontal cortex. (D) Analysis of mGluR5 and beta-arrestin levels in the cytoplasmic fraction of the frontal cortex. * Indicates a significant difference between alpha-syn tg mice and non-tg controls p<0.05, one-way ANOVA and post hoc Fisher). # Indicates a significant difference between PDGF-alpha-syn and mThy1-alpha-syn tg mice (p<0.05, one-way ANOVA and post hoc Fisher)(n = 8 mice per group).

### mGluR5 interacts with α-syn in the brains of transgenic animals

In order to identify whether the alterations in mGluR5 protein levels were related to transcription changes at the mRNA level, qPCR analysis was conducted. By qPCR, levels of mRNA were comparable between DLB, PD and control cases (Figure S3A) non-tg and PDGF- and mThy1-alpha-syn tg mice (Figure S3B), suggesting that transcriptional events are not involved and that the interaction between alpha-syn and mGluR5 occurs post-transcription/post-translationally. Since, mGluR5 alterations by immunoblot were primarily detected in the membrane rather than cytosolic fractions and were accompanied by increased expression of beta-arrestin suggesting that mGluR5 localization might be altered by alpha-syn. Immunohistochemical double labeling with antibodies against alpha-syn and mGluR5 showed a small degree of alpha-syn co-localization with mGluR5 within the frontal cortex of controls (Figure 5A-C) however the degree of co-localization was greatly increased in the DLB (Figure 5D–F) and PD (Figure 5G–I) cases. Consistent with the human cases, non-tg mice showed a small degree of alpha-syn co-localization with mGluR5 within pyramidal neurons in the frontal cortex of (Figure 5J–L) however the degree of co-localization was greatly increased in the PDGF-alpha-syn tg (Figure 5M–O) and mThy1-alpha-syn tg (Figure 5P–R) mice.

**Figure 5:** Co-immunoprecipitation and co-localization of alpha-syn and mGluR5. (A, D, G) Representative confocal images of alpha-syn immunolabeling in the frontal cortex of control, DLB and PD cases, respectively. (B, E, H) Representative confocal images of mGluR5 immunolabeling in the frontal cortex of control, DLB and PD cases, respectively. (C, F, I) Co-localization of alpha-syn and mGluR5 immunoreactivity in the frontal cortex of control, DLB and PD cases, respectively. (J, M, P) Representative confocal images of alpha-syn immunolabeling in the frontal cortex of non-tg, PDGF-alpha-syn tg and mThy1-alpha-syn tg mice, respectively. (K, N, Q) Representative confocal images of mGluR5 immunolabeling in the frontal cortex of non-tg, PDGF-alpha-syn tg and mThy1-alpha-syn tg mice, respectively. (L, O, R) Co-localization of alpha-syn and mGluR5 immunoreactivity in the frontal cortex of non-tg, PDGF-alpha-syn tg and mThy1-alpha-syn tg mice, respectively. (S) Representative immunoblot of the co-immunoprecipitation of mGluR5 and alpha-syn using the anti-mGluR5 antibody for the pull-down and the alpha-syn antibody for the detection. (T) Representative immunoblot of the co-immunoprecipitation of mGluR5 and alpha-syn using the alpha-syn antibody for the pull-down and the anti-mGluR5 antibody for the detection. Scale bar  = 20 µM.

In order to examine whether mGluR5 and alpha-syn interact (directly or indirectly) co-immunoprecipitation (co-IP) studies were conducted. When samples from the mouse brains of non-tg, PDGF-alpha-syn and mThy1-alpha-syn tg mice were immunoprecipitated with an antibody against mGluR5 and then analyzed by immunoblot with an antibody against alpha-syn, the strongest interaction was observed in the alpha-syn tg mice when compared to non-tg controls (Figure 5S). No interacting bands were detected in control experiments with samples immunoprecipitated with a non-immune IgG or when the tissue sample was excluded. Similarly when the reverse IP was performed, by immunoprecipitating with an antibody against alpha-syn and then analyzing by immunoblot with an antibody against mGluR5, the strongest interaction was again observed in the alpha-syn tg mice when compared to non-tg controls (Figure 5T). No interacting bands were detected in control experiments with samples immunoprecipitated with a non-immune IgG. To further validate the IP, samples immunoprecipitated with the antibody against alpha-syn were analyzed with an antibody against alpha-syn. This study confirmed that in the samples from the alpha-syn tg mice higher levels of alpha-syn immunoreactivity were detected than in the non-tg mice (data not shown).

### Wide field mosaic analysis of alpha-syn and mGluR5 distribution in alpha-syn transgenic mice

Wide field mosaic imaging was conducted to examine in a more comprehensive manner the relationship between the distribution of alpha-syn and mGluR5 immunolabeling in several brain regions associated with rodent spatial memory and motor functions. (Figure S4). Patterns of alpha-syn and mGluR5 immunolabeling were examined within the motor cortex, piriform cortex, four sub-regions of striatum, three regions within the hippocampal formation, and the substantia nigra. Alpha-syn immunolabeling in non-tg samples was punctate in nature, and no labeled cell bodies or neurites were observed in any samples. In contrast, alpha-syn immunolabeling in tg mice was noticeably increased, more diffuse in nature, and immunopositive cell bodies, dendrites and other elements in the neuropil were observed in many regions. In comparison, increased mGluR5 immunolabeling was noted in nearly identical regions. The regional statistics are provided in Table 2. Within the motor cortex (Figure S4B) an increase in alpha-syn was noted in tg versus non-tg samples.

**Table 2:** Regional statistics and percentages for α-syn and mGluR5 immunolabeling for data presented in Figure S4.

*Mouse CNS region*	*alpha-syn Immunolabeling*	*mGluR5 Immunolabeling*
*Motor Cortex*	*+95.7%* *p*<0.05, F(1,11) = 8.99	*+120.8%* *p*<0.01, F(1,11) = 20.64
*Piriform Cortex*	*+5.6%*n.s., F(1,9) = 0.28	*+53.13%* *P*<0.01, F(1,9) = 51.59
*Dorsomedial Striatum*	*+275.6%* *p*<0.01, F(1,14) = 17.60	*+159.6%* *p*<0.01, F(1,14) = 55.63
*Dorsolateral Striatum*	*+199.6%* *p*<0.01, F(1,14) = 17.22	*+150.6%* *p*<0.01, F(1,14) = 100.54
*Ventromedial Striatum*	*+42.7%* *p*<0.05, F(1,14) = 8.57	*+62.3%* *p*<0.05, F(1,14) = 4.77
*Ventrolateral Striatum*	*+112.2%* *p*<0.01, F(1,14) = 8.04	*+98.5%* *p*<0.01, F(1,14) = 38.27
*Substantia Nigra*	*+55.5%* *p*<0.01, F(1,11) = 7.41	*+59.26%* *p*<0.05, F(1,11) = 7.41
*CA1 region*	*+178.5* *p*<0.01, F(1,10) = 103.95	*+51.52%*n.s., F(1,10) = 4.57
*CA3 region*	*+97.8%* *p*<0.05, F(1,7) = 8.97	*+259.3%* *p*<0.01, F(1,7) = 42.53
*Dentate Gyrus*	*+51.4%* *p*<0.05, F(1,17) = 6.70	*+80.7%* *p*<0.01, F(1,17) = 32.59

The mGluR5 labeling was diffuse in nature and included immunopositive cell bodies present within the inner granular cell layer. In non-tg samples we observed apparent axonal mGluR5 immunolabeling through the cortical layers presumably on pyramidal cell axons. This pattern was also seen in the tg samples, with a noticeable increase in the amount of staining, as well as an extension of staining to varicosities along the axonal projections through the outer granular layer. Alpha-syn immunolabeling within tg piriform cortex (Figure S4B, C) was also more diffuse, with immunopositive cell bodies and neurites present within the cell body layers II and III. mGluR5 immunolabeling within the piriform cortex of non-tg animals consisted of punctate staining throughout the cell body layer. The levels were increased in tg samples and also included increased axonal staining through the piriform cortical cell body layers II and III. In contrast with the immunostaining patterns observed within the aforementioned cortical regions, the pattern of alpha-syn immunolabeling within tg striatal regions (dorsomedial, dorsolateral, ventromedial and ventrolateral) was punctate, and synaptic like in nature. No immunopositive cell bodies or neurites were observed in any striatal region (Figure S4B, D). Striatal mGluR5 immunolabeling in tg samples was increased within the neuropil, and also included perineuronal staining not observed in the non-tg. Sparse, small, punctate alpha-syn immunolabeling was found in the substantia nigra pars compacta (SNc) in non-tg samples. SNc immunolabeling was increased in tg samples, with the addition of tyrosine hydroxylase-like labeled projections innervating the substantia nigra pars reticulata (Figure S4B). mGluR5 immunolabeling was increased in the SNc and consisted of labeled fibers and neurites, in a pattern similar to TH immunoreactivity.

Within the hippocampal formation we examined alpha-syn and mGluR5 immunolabeling within CA1, CA3 and dentate gyrus. Within the CA1 field of non-tg samples, alpha-syn immunolabeling within the neuropil was largely confined to the area immediately surrounding the pyramidal cell layer. Within the pyramidal cell layer of CA1, alpha-syn immunolabeling was present on axonal projections and surrounding cell bodies. mGluR5 labeling within the CA1 largely followed the pattern of alpha-syn immunoreactivity. Axonal mGluR5 staining was also evident through the extent of the pyramidal cell layer with labeled axonal projections towards the stratum radiatum (Figure S4B). Within the CA3 region of non-tg samples, punctate alpha-syn immunolabeling was largely confined to the area adjacent to the stratum lucidum. An expansion of alpha-syn immunoreactivity was seen in tg samples with an increase in staining within the neuropil, and including many immunopositive cell bodies within the stratum lucidum (Figure S4B). In non-tg samples, the pattern of larger punctate mGluR5 immunolabeling corresponded to the distribution of alpha-syn immunoreactivity. Like alpha-syn immunoreactivity in tg animals, mGluR5 immunolabeling was increased in tg mice throughout the neuropil and surrounded cell bodies within the stratum lucidum.

Alpha-syn immunolabeling was sparse within all sub-regions of non-tg dentate gyrus, and was substantially increased within molecular layers, hilus and supra- and infrapyramidal blades of the dentate gyrus (Figure S4B). This included punctate labeling in the neuropil surrounding cell bodies and cytoplasmic labeling of cells within the hilus. mGluR5 labeling of non-tg dentate gyrus included labeling of collateral varicosities within the hilus, diffuse labeling of the neuropil in the molecular layers, and minimal axonal-like labeling through cell body layers of the suprapyramidal and infrapyramidal blades. The intensity of mGluR5 labeling was increased in tg samples and included labeling of intracytoplasmic regions of large neuronal cell bodies, with an approximate shape and size appropriate for interneurons and main apical dendrites within the hilus.

### Increased mGluR5 signaling in DLB/PD and alpha-syn transgenic mice

In order to investigate whether the increased mGluR5 level in the DLB and PD cases and in the alpha-syn tg mice was associated with a concomitant increase in the levels of downstream signaling components, levels of total and phosphorylated ERK, Elk–1 and CREB were examined in the cytoplasmic and membrane fractions from the frontal cortex. In the membrane fraction ERK activation (ratio of pERK/tERK) was increased in the DLB and PD cases in comparison to the control cases (Figure 6A, E). Elk-1 activation (ratio of pElk-1/tElk-1) was increased in the membrane fraction from the DLB cases but not PD cases, when compared to controls. (Figure 6A, G). CREB activation (ratio of pCREB/tCREB) was increased in the nuclear fraction from the DLB and PD cases when compared to controls (Figure 6C, I), In the cytoplasmic fraction, both DLB and PD cases displayed increased ERK activation (ratio pERK/totalERK) compared to control cases (Figure 6B, F). No significant differences in Ekl-1 activation were noted between DLB or PD cases and controls (Figure 6B, H). CREB activation was decreased in the soluble fraction from both DLB and PD when compared to control cases (Figure 6D, J). A similar immunoblot to investigate downstream signaling components was conducted on the membrane, cytosolic and nuclear fractions from the frontal cortex of non-tg and alpha-syn tg mice (Figure 7).

**Figure 6:** Immunoblot analysis of ERK, Elk-1 and CREB activity in Control, DLB and PD cases. (A) Representative immunoblot of phospho-ERK (pERK), total ERK (tERK) phospho-ELK-1 (pELK-1) and total ELK-1 (tELK-1) expression levels in the membrane fraction from the frontal cortex of control, DLB and PD cases. (B) Representative immunoblot of pERK, tERK, pELK-1 and tELK-1 expression in the cytoplasmic fraction from the frontal cortex of control, DLB and PD cases. (C) Analysis of ERK activity (pERK/tERK ratio) in the membrane fraction. (D) Analysis of ERK activity (pERK/tERK ratio) in the cytosolic fraction. (E) Analysis of Elk-1 activity (pElk-1/tElk-1 ratio) in the membrane fraction. (F) Analysis of Elk-1 activity (pElk-1/tElk-1 ratio) in the cytosolic fraction. (G) Representative immunoblot of phospho-CREB (pCREB) and total CREB (tCREB) in the nuclear fraction from the frontal cortex of control, DLB and PD cases. (H) Representative immunoblot of pCREB and tCREB in the soluble fraction from the frontal cortex of control, DLB and PD cases. (I) Analysis of CREB activity in the nuclear fraction. (J) Analysis of CREB activity in the soluble fraction. * Indicates a significant difference between DLB or PD cases compared to control cases. (p<0.05, one-way ANOVA and post hoc Fisher) (n = 8 cases per group).

**Figure 7:** Immunoblot Analysis of ERK, Elk-1 and CREB activity in alpha-syn transgenic mice. (A) Representative immunoblot of phospho-ERK (pERK), total ERK (tERK) phospho-ELK-1 (pELK-1) and total ELK-1 (tELK-1) expression levels in the membrane fraction from the frontal cortex of non-tg, PDGF-alpha-syn and mThy1-alpha-syn tg mice. (B) Representative immunoblot of pERK, tERK, pELK-1 and tELK-1 expression in the cytoplasmic fraction from the frontal cortex of non-tg, PDGF-alpha-syn and mThy1-alpha-syn tg mice. (C) Analysis of ERK activity (pERK/tERK ratio) in the membrane fraction. (D) Analysis of ERK activity (pERK/tERK ratio) in the cytosolic fraction. (E) Analysis of Elk-1 activity (pElk-1/tElk-1 ratio) in the membrane fraction. (F) Analysis of Elk-1 activity (pElk- 1/tElk-1 ratio) in the cytosolic fraction. (G) Representative immunoblot of phospho- CREB (pCREB) and total CREB (tCREB) in the nuclear fraction from the frontal cortex of non-tg, PDGF-alpha-syn and mThy1-alpha-syn tg mice. (H) Representative immunoblot of pCREB and tCREB in the soluble fraction from the frontal cortex of non-tg, PDGF-alpha-syn and mThy1-alpha-syn tg mice. (I) Analysis of CREB activity in the nuclear fraction. (J) Analysis of CREB activity in the soluble fraction. * Indicates a significant difference between alpha-syn tg mice and non-tg controls p<0.05, one-way ANOVA and post hoc Fisher). # Indicates a significant difference between PDGF-alpha-syn and mThy1-alpha-syn tg mice (p<0.05, one-way ANOVA and post hoc Fisher)(n = 8 mice per group).

The ERK activation was increased in the mThy-1-alpha-syn tg mice in both the membrane (Figure 7A, E) and cytoplasmic (Figure 7B, F) fractions in comparison to non-tg controls, however it did not differ between PDGF-alpha-syn tg mice and non-tg controls on either fraction (Figure 7A, B, E, F). The membrane fraction both the PDGF-alpha-syn and mThy1-alpha-syn tg mice displayed increased levels of Elk-1 activation in comparison to non-tg controls (Figure 7A, G). No Elk-1 activation was detected in the cytoplasmic fraction (Figure 7B, H). CREB activation was increased in the PDGF-alpha-syn and mThy1-alpha-syn tg mice in the nuclear fraction compared to non-tg controls (Figure 7C, I), however in the soluble fraction CREB activation was only increased in the mThy1-alpha-syn tg mice when compared to non-tg controls (Figure 7D, J).

### Motor deficits in the pole test apparatus in alpha-syn transgenic mice are ameliorated by the mGluR5 inhibitor MPEP

In the tg mice there is considerable accumulation of alpha-syn in the caudo-putamen region that is accompanied by motor deficits in the pole test. Since it is possible that increased expression of mGluR5 in mid-spine neurons as shown here might play a role in the motor deficits, non-tg and alpha-syn tg mice were treated with the mGluR5 antagonist MPEP and tested in the pole test. This behavioral test requires the subjects to grip and traverse the pole requiring motor strength and coordination [54], [63]. The stringent test parameters help to ensure that tg deficits are not obscured by compensatory responses (*e.g.* incomplete turns prior to descending the pole apparatus). Compared with non-tg mice, alpha-syn tg mice were impaired in ability to negotiate the pole apparatus as evidenced by a significant longer T-Turn time (Baseline, Figure 8A).

**Figure 8:** Motor and learning/memory deficits in alpha-syn transgenic mice are ameliorated by MPEP administration. (A) Pole test performance (T-Turn) of the non-tg and PDGF-alpha-syn tg mice, at baseline, following MPEP treatment and at re-test (no treatment). (B) Morris water maze performance of vehicle-treated non-tg and PDGF-alpha-syn tg mice. (C) Morris water maze performance of MPEP- treated PDGF-alpha-syn tg mice. (D) Morris water maze performance of MPEP-treated non-tg mice. * Indicates a significant difference between groups examined (p<0.05, one-way ANOVA and post hoc Fisher) (n = 8 per group).

To assess whether mGluR5 antagonism could ameliorate the pole test behavioral deficit observed in the tg animals, mice were treated with the mGluR5 antagonist MPEP. Following treatment with MPEP T-Turn was comparable between the non-tg and alpha-syn tg mice (MPEP Treatment, Figure 8A). Analysis of the difference between the first and second test days revealed an improvement in T-Turn times of the alpha-syn tg mice as indicated by significant improvement in the success ratio from the first test to second test session (F(1,6) = 6.40; p = 0.0447). When the mice were tested a day after the MPEP treatment (Re-test, no treatment, Figure 8A), once more alpha-syn tg mice displayed impaired performance in the pole test when compared to the non-tg controls (F(1,6) = 18.498; p = 0.0051).

### The spatial memory deficits in alpha-syn transgenic mice are ameliorated by the mGluR5 inhibitor MPEP

Though motor deficits are more often highlighted, cognitive deficits associated with alpha-syn accumulation in the limbic system have also been reported in patients with Parkinson's disease dementia and dementia with LB's [56]. These alterations might be associated with the increased expression of mGluR5 in the frontal cortex and hippocampus of the alpha-syn tg mice. To investigate this possibility, mice were tested in the water maze and treated with the mGluR5 antagonist MPEP. During the training period of the test, repeated measures ANOVA revealed no significant differences among the groups path length (F(1,12) = 2.294, p = 0.1557 and F(1,6) = 0.500, p = 0.8060). During the spatial learning period of the test with the platform submerged, vehicle treated alpha-syn tg mice displayed performance deficits when compared to the vehicle treated non-tg controls (Figure 8B). In contrast, MPEP treatment improved the behavioral performance of the alpha-syn tg compared to the vehicle treated alpha-syn tg mice (Figure 8C). The MPEP treated alpha-syn tg mice performance was similar to the non-tg controls. In the last day of testing the platform was removed. The probe test indicated a significant main effect of the genotype on entrances and passes into target zone (F(1,12) = 6.649, p = 0.0242). In contrast, alpha-syn tg mice treated with MPEP exhibited a similar number of entrances and passes into target zone when compared to the non-tg controls. MPEP treatment had no effect on the performance of the non-tg mice (Figure 8D).

A subsequent trial in which the platform was visible, confirmed that both groups were able to locate the platform via visual sighting. These results indicate that the deficit in ability to locate the correct zone, seen in the alpha-syn tg mice, is not attributable to a visual or gross motor deficit, but is instead likely to be a consequence of a memory or spatial navigation defect.

## Discussion

Excitoxicity has been proposed to play a role in the mechanisms of neurodegeneration in DLB and PD. The present study showed that alterations in the levels of mGluR5 in selected brain regions in patients with DLB or PD and in alpha-syn transgenic mice might be involved. Specifically, mGluR5 was increased in the frontal cortex, hippocampus and caudate in DLB in and in the caudate in PD, these areas correspond closely with areas displaying increased alpha-syn accumulation. The results of this study are consistent with previous studies that have shown increased expression or activation of glutamate receptors in the acute neurotoxicity rodent [43] and primate [64] models of PD and in other neurodegenerative disorders with protein accumulation such as Amyotrophic lateral sclerosis (mGluR5; [65]), Down's syndrome (mGluR5; [66]), and AD (mGluR2/3; [32], [67], [68], [69]). However, our study is the first to document alterations in mGluR5 in human DLB and PD cases and in alpha-syn tg mice.

The important of metabotropic glutamate receptors, particularly mGluR5, in neurodegenerative disorders is underlined by recent work suggesting that excitotoxicity mediated by metabotropic receptors may be a key mechanism underlying neurodegeneration [70], [71] and by recent experimental therapies based in the development of mGluR5 antagonists [71], [72], [73], [74]. Consistent with this proposed role of mGluR5 in excitotoxicity and the potential therapeutic use of mGluR5 antagonists we show that when the alpha-syn tg mice were treated with the mGluR5 antagonist MPEP their motor and learning/memory deficits were ameliorated. This is in agreement with previous studies showing that mGluR5 inhibitors reduce the motor alterations in rodent models challenged with MPTP or 6-OH DOPA [75], [76], [77], [78] and recent studies in primates showing that MPEP and another mGluR5 antagonist such as MTEP (3-((2-Methyl-4-thiazolyl)ethynyl)pyridine) has beneficial anti-dyskinetic effects in L-Dopa-treated MPTP monkeys [79], [80]. Moreover, co-administration of adenosine 2A and mGluR5 antagonists reverses the behavioral deficits in a reserpinized mouse model of PD [51]. In addition to the effects at reducing motor alterations, MPEP has been shown to reduce the visuo-spatial discrimination deficit induced by bilateral dopamine lesion of the striatum [81]. This same treatment increased contralateral turning induced by L-DOPA in mice bearing unilateral 6-OHDA lesion suggesting that mGluR5 blockade may also have beneficial effects on cognitive deficits induced by dopamine depletion [81]. Therefore, both neurotoxic and transgenic models of parkinsonism support the possibility that antagonism of mGluR5 might be potentially beneficial in the treatment of DLB and PD patients.

mGluR5 has attracted considerable interest due to its abundant expression in the frontal cortex, limbic system, and caudo-putamen [37]—brain regions selectively affected in PD. The vulnerability of selected neuronal populations in PD and DLB patients has been linked to glutamate-mediated excitotoxicity [82]. Consistent with this, the double labeling and mosaic analysis showed that there was some regional specificity to the increased levels of mGluR5 that corresponded to the areas of greater α-syn accumulation and neurodegeneration. For example, in the DLB cases mGluR5 was elevated in the frontal cortex, limbic system and putamen, while in the PD cases the increase was more prominent in the putamen. In the PDGF-alpha-syn tg mice mGluR5 increases were more prominent in the frontal cortex and limbic system while in the mThy1-alpha-syn tg mice mGluR5 was also elevated in the striatum. Of the affected areas mGluR5 was found in pyramidal neurons in the deeper layers of the frontal cortex, CA3 region of the hippocampus and mid-spiny neurons in the striatum. These are all neuronal populations and brain regions selectively affected in DLB and PD patients [11], [83], [84], [85] suggesting that mGluR5 might play a role in the mechanisms of selective neuronal vulnerability in disorders with alpha-syn accumulation.

The precise mechanisms by which alpha-syn accumulation in DLB, PD and tg models might lead to the increase mGluR5 is not completely clear. However the alterations in mGluR5 are most likely post-translational since levels of mGluR5 mRNA did not differ between control and DLB or PD cases or between non-tg and alpha-syn transgenic mice. Thus, it is possible that alpha-syn interacts with mGluR5 to alter the distribution of these receptors at the cell membrane of particular cell populations, which may lead to an increase in mGluR5 activity and glutamate-mediated excitotoxicity in specific brain regions. In support of this interaction hypothesis we showed a greater degree of mGluR5 and alpha-syn co-immunoprecipitation in the alpha-syn tg mice compared to non-tg mice and a greater accumulation of mGluR5 in the membrane fractions from DLB or PD cases and in alpha-syn tg mice compared to control cases or non-tg mice. Moreover the increase in mGluR5 was accompanied by an increase in beta-arrestin, a protein involved in the internalization and recycling of the receptor. Taken together, these results suggest that accumulation of alpha-syn might alter mGluR5 localization at the cell surface, allowing a greater proportion to remain membrane-associated rather than being recycled.

If this is the case, then it is also possible that increased presence of the receptor at the cell surface may lead to over activation of the downstream mGluR5 signaling pathway. mGluR5 is a Group I metabotropic glutamate receptor that couples with phospholipase C (PLC) via Gq-like G-proteins. PLC activates protein kinase-C (PKC) activation via diacylglycerol and PKC goes on to phosphorylate and activate ERK, which activates ElK-1. PLC additionally activates inositol 1,4,5-trisphosphate (IP3) resulting in the release of calcium from intracellular stores such as the endoplasmic reticulum. This calcium in turn activates a number of calcium-responsive proteins such as those involved in the calcium/calmodulin/calmodulin kinase (CaM kiinase) cascade including CaMKinase I and IV which phosphorylate cyclic-AMP response element-binding (CREB) and activate gene expression [86].

We demonstrate that the increased expression of mGluR5 in DLB, PD and alpha-syn tg mice is accompanied by an increase activation of down-stream signaling pathway components including ERK, Elk-1 and CREB. Dysregulated calcium homeostasis has been linked to a number of neurodegenerative diseases including PD and AD [87] and as over activation of the mGluR5 signaling pathway may also contribute to increases in intracellular calcium it might play a role in mGluR5-mediated selective vulnerability.

In addition to the increased expression and over activation of mGluR5, alpha-syn has been reported to interact with individual components of the mGluR5 signaling pathway including ERK and Elk-1 [88], [89], this is supported by the detection of ERK, Elk-1 and alpha-syn in Lewy Body aggregates. Iwata and colleagues have demonstrated that in vitro over expression of alpha-syn reduces ERK-1/2 phosphorylation and activation of ERK-1/2 signaling, eventually resulting in cell death [90]. Therefore it is possible that alpha-syn may modulate mGluR5 activity both directly - by increasing cell surface concentrations of the receptor itself, as evidenced by the concomitant increase in levels of beta-arrestin that may serve to keep greater proportions of the receptor at the cell surface rather than being recycled and indirectly - by binding to the downstream signaling components of the mGluR5 pathway.

Taken together the results from study this support the notion that alpha-syn may directly interact with mGluR5 resulting in its over activation and suggest that this over activation may contribute to excitotoxic cell death in selected neuronal populations expressing higher levels of mGluR5. These results also highlight the potential therapeutic importance of mGluR5 antagonists in disorders characterized by alpha-syn accumulation.

## Supporting Information

Figure S1 Hippocampal and caudate levels of mGluR5 in Control, DLB and PD cases. (A–C) Representative images of mGluR5 immunoreactivity in the CA2/3 of the hippocampus from control, DLB and PD cases respectively, analyzed in (D). (E–G) Representative images of mGluR5 immunoreactivity in the caudate from control, DLB and PD cases respectively, analyzed in (H). Scale bar  = 50 µM * Indicates a significant difference between DLB or PD cases compared to control cases (p<0.05, one-way ANOVA and post hoc Fisher). # Indicates a significant difference between DLB and PD cases (p<0.05, one-way ANOVA and post hoc Fisher) (n = 8, case per group).
(2.38 MB TIF)

Figure S2 Hippocampal and caudate levels of mGluR5 in alpha-syn transgenic mice. (A–C) Representative images of mGluR5 immunoreactivity in the CA2/3 of the hippocampus of non-tg, PDGF-alpha-syn and mThy1-alpha-syn tg mice respectively, analyzed in (D). (E–G) Representative images of mGluR5 immunoreactivity in the caudate of non-tg, PDGF-alpha-syn and mThy1-alpha-syn tg mice respectively, analyzed in (H). * Indicates a significant difference between alpha-syn tg mice compared to non-tg controls (p<0.05, one-way ANOVA and post hoc Fisher).
(2.34 MB TIF)

Figure S3 mGluR5 mRNA levels in Control, DLB and PD cases and alpha-syn transgenic mice. (A) Quantitative real-time PCR (qPCR) analysis of mGluR5 mRNA levels in Control, DLB and PD cases. (B) qPCR analysis of mGluR5 mRNA levels in non-tg, PDGF-alpha-syn tg and mThy1-alpha-syn tg mice.
(0.27 MB TIF)

Figure S4 High-resolution, large-scale maps of alpha-syn and mGluR5 in alpha-syn transgenic mice. (A) Representative confocal image depicting localization of alpha-syn (green) and mGluR5 (red) immunoreactivity in an alpha-syn tg mouse brain - inset at higher magnification in the right panel. (B) Representative confocal image depicting localization of alpha-syn and mGluR5 immunoreactivity in the motor cortex (mCtx), piriform cortex (pCtx), CA1 region of hippocampus (CA1), CA3 region of hippocampus, (CA3), dentate gyrus (DG), dorsomedial striatum, (dmSTR) and substantia nigra (SN) in non-tg and alpha-syn tg mice respectively. (C) Semi-quantitative analysis of mGluR5 immunoreactivity in the mCtx, pCtx, CA1, CA3, and DG of non-tg and alpha-syn tg mice. (D) Semi-quantitative analysis of mGluR5 immunoreactivity in the dmSTR, dorsolateral striatum (dlSTR), ventromedial striatum (vmSTR), ventrolateral striatum (vlSTR) and SN of non-tg and alpha-syn tg mice. Imaging parameters were kept consistent within regions and data are presented as mean pixel intensity ± SEM. * Indicates a significant difference between non-tg and alpha-syn tg mice (p<0.05, one-way ANOVA and post hoc Fisher).
(5.47 MB TIF)
